# MeCP2‐421‐mediated RPE epithelial‐mesenchymal transition and its relevance to the pathogenesis of proliferative vitreoretinopathy

**DOI:** 10.1111/jcmm.15602

**Published:** 2020-07-08

**Authors:** Xiaohua Li, Xue Li, Shikun He, Mingwei Zhao

**Affiliations:** ^1^ Henan Provincial People's Hospital Zhengzhou China; ^2^ Henan Eye Hospital Henan Eye Institute Henan Key Laboratory of Ophthalmology and Visual Science Zhengzhou China; ^3^ People's Hospital of Zhengzhou University Zhengzhou China; ^4^ People's Hospital of Henan University Zhengzhou China; ^5^ Ophthalmology Optometry Centre Peking University People's Hospital Beijing Key Laboratory of Diagnosis and Therapy of Retinal and Choroid Diseases Beijing China; ^6^ Departments of Pathology USC Roski Eye Institute, Keck School of Medicine University of Southern California Los Angeles CA USA

**Keywords:** EMT, P‐MeCP2‐421, PVR, RPE, TGF‐β

## Abstract

Proliferative vitreoretinopathy (PVR) is a blinding eye disease. Epithelial‐mesenchymal transition (EMT) of RPE cells plays an important role in the pathogenesis of PVR. In the current study, we sought to investigate the role of the methyl‐CpG‐binding protein 2 (MeCP2), especially P‐MeCP2‐421 in the pathogenesis of PVR. The expressions of P‐MeCP2‐421, P‐MeCP2‐80, PPAR‐γ and the double labelling of P‐MeCP2‐421 with α‐SMA, cytokeratin, TGF‐β and PPAR‐γ in human PVR membranes were analysed by immunohistochemistry. The effect of knocking down MeCP2 using siRNA on the expressions of α‐SMA, phospho‐Smad2/3, collagen I, fibronectin and PPAR‐γ; the expression of α‐SMA stimulated by recombinant MeCP2 in ARPE‐19; and the effect of TGF‐β and 5‐AZA treatment on PPAR‐γ expression were analysed by Western blot. Chromatin immunoprecipitation was used to determine the binding of MeCP2 to TGF‐β. Our results showed that P‐MeCP2‐421 was highly expressed in PVR membranes and was double labelled with α‐SMA, cytokeratin and TGF‐β, knocking down MeCP2 inhibited the activation of Smad2/3 and the expression of collagen I and fibronectin induced by TGF‐β. TGF‐β inhibited the expression of PPAR‐γ, silence of MeCP2 by siRNA or using MeCP2 inhibitor (5‐AZA) increased the expression of PPAR‐γ. α‐SMA was up‐regulated by the treatment of recombinant MeCP2. Importantly, we found that MeCP2 bound to TGF‐β as demonstrated by Chip assay. The results suggest that MeCP2 especially P‐MeCP2‐421 may play a significant role in the pathogenesis of PVR and targeting MeCP2 may be a potential therapeutic approach for the treatment of PVR.

## 1 INTRODUCTION

One of serious complications of ocular trauma and failed repair of primary rhegmatogenous retinal detachment is proliferative vitreoretinopathy (PVR).^1^, ^2^, ^3^ PVR is an exaggerated wound healing process and a major cause of vision loss due to trauma. The essential pathogenesis of PVR is poorly understood, and there is no effective cure or prevention of PVR, so the loss of vision due to PVR has a serious socioeconomic effect.

Although inflammatory cells and glial cells participate in the formation of PVR, it is known that retinal pigment epithelium (RPE) cells are the key player in the pathogenesis of PVR.^1^, ^2^, ^3^ In PVR, RPE cells are undergone epithelial‐mesenchymal transition (EMT) and differentiate into a myofibroblast phenotype cell that migrates and proliferates to form retinal fibrotic membranes,^4^, ^5^, ^6^, ^7^, ^8^ and a variety of inflammatory cytokines, numerous growth factors (particular TGF‐β) and extracellular matrix (ECM) are involved in the pathogenesis of PVR ^9^, ^10^, ^11^, ^12^, ^13^; however, limited knowledge is known about the basic mechanisms of PVR development. Understanding of the cause and progression of PVR is needed to support development of new therapeutic strategies based on a mechanistic understanding of the disease.

It is known that TGF‐β is the major inducer of EMT and retinal fibrosis.^7^, ^10^, ^11^ TGF‐β binds its receptor and activates Smad2/3 signalling and regulates several transcription factors that mediate the expression of α‐SMA and ECM such as collagen and fibronectin (FN) deposition and fibrosis.^12^, ^13^, ^14^, ^15^ In addition, increased TGF‐β activity is associated with the down‐regulation of the genes of trans‐differentiation inhibitor such as peroxisome proliferator–activated receptor‐γ (PPAR‐γ),^16^, ^17^ which is a key negative regulator of TGF‐β signalling. Inhibition of TGF‐β signalling via knocking down Smad2/3 has been demonstrated to suppress the expression of α‐SMA, collagen and experimental PVR in mice.^12^, ^13^

Recent studies suggest that wound healing process including fibrosis is also regulated by epigenetic factors including the factors of DNA methylation, histone modification ^18^, ^19^, ^20^, ^21^ and non‐coding RNA; specifically, the methyl‐CpG‐binding protein 2 (MeCP2) has been demonstrated to play a pivotal role in fibrosis of systemic diseases.^19^, ^22^, ^23^, ^24^, ^25^ MeCP2 binds to methylated DNA and has been considered as a classic epigenetic factor that regulates gene expression. In a rat liver fibrosis model, MeCP2 expression is predominately associated with myofibroblastic cells and was found to selectively expressed in fibrotic tissues ^19^; however, in non‐trans‐differentiated cells MeCP2 expression is low,^19^, ^22^ and furthermore, MeCP2 acts as powerful epigenetic regulator for the genes related to myofibroblast trans‐differentiation, knocking down MeCP2 by siRNA increases the expression of PPAR‐γ.^19^, ^22^ Cell migration is also inhibited by silencing MeCP2.^21^ The expression of MeCP2 is regulated by a number of factors.^26^ There are many sites of serine phosphorylation in MeCP2 molecular; notably, most known MeCP2 that mediated gene activation is related to its phosphorylation at Serin421,^27^, ^28^, ^29^, ^30^, ^31^ and it is known that phosphorylation of MeCP2 leads to its dissociation with sin3 and HDAC and gene activation.^32^ Therefore, MeCP2 not only functions as a transcription repressor, but also acts as gene expression activator.^27^, ^31^, ^32^, ^33^ Although the expression of MeCP2 in PVR membranes has been reported,^21^ the relevance of its phosphorylation especially P‐MeCP2‐421 PVR remained unclear. In the current study, we sought to investigate the role of P‐MeCP2‐421 in the pathogenesis of PVR.

## 2 PATIENTS AND METHODS

All procedures conformed to the Declaration of Helsinki for research involving human subjects. The Institutional Review Board of Henan Eye Institute approved the use of human specimens. Informed consent was obtained from all individuals. Retinal sections from patients with PVR 10 eyes and retinal sections from the eyes without PVR (6 eyes) were included in the study. The medical records of all patients were reviewed retrospectively. The PVR membranes were obtained from the patients with PVR who had undergone pars plana vitrectomy and membrane peeling by retinal specialist in our eye hospital. Patients who had received intraocular injections of steroids or any other drugs before surgery were excluded.

### 2.1 Immunohistochemistry

The surgically excised PVR membranes from the patients were fixed in 4% paraformaldehyde, and 3‐µm paraffin sections were obtained. The methods of the details of the Immunohistochemistry were described before.^27^ Briefly, antigen retrieval was performed and the tissue section was blocked with 5% normal goat serum for 30 minutes. Anti‐phosphorylated MeCP2‐S80 (Thermo Fisher Scientific) and anti‐phosphorylated MeCP2‐S421 (ABGENT) were applied to the sections for 1 hour in room temperature and then followed by biotinylated secondary anti‐rabbit antibody (1:400; Vector Laboratories) and streptavidin peroxidase for 30 minutes, respectively. Between each step, the slides were washed three times with PBS (PH.7.2). An aminoethyl carbazole kit (Zymed) was used to detect the immunoreactivity. Isotype‐matched primary antibody was used as a negative control. Haematoxylin was applied to the slides for contrast staining. Retinal sections from patients with eyelid tumour orbital extension who underwent exenteration were used as control.

### 2.2 Immunofluorescence double labelling

For double labelling, anti‐phospho‐MeCP2‐421 antibodies were applied to the sections and incubated at 4°C overnight. Next day, a rhodamine‐conjugated secondary antibody (red colour) was used for additional 30‐minutes incubation. After washing with PBS, the sections were incubated with the antibodies specific for a‐SMA (monoclonal mouse anti‐a‐SMA, 1:100 dilution, clone 1A4; Sigma‐Aldrich Corp.), cytokeratin (Abcam), TGF‐β (Santa Cruz Biotechnology) and PPAR‐γ (Biosis) for 1 hour. The sections were washed again with PBS and then incubated with secondary antibody conjugated to fluorescein isothiocyanate for 30 minutes. After PBS washing, the slides were mounted with Hoechst mounting medium (Solarbio). The double labelling was observed by confocal laser‐scanning microscopy (Nikon C1 Si). Isotype‐matched primary antibody was used for negative controls.

### 2.3 Cell culture and treatment

Human ARPE‐19 cells were obtained from ATCC (Manassas, VA) and were maintained culture in DMEM with addition of 2 mmol/L L‐glutamine, 100 U/mL penicillin, 100 μg/mL streptomycin (Sigma‐Aldrich) and 10% foetal bovine serum (FBS; Irvine Scientific, Santa Ana, CA). The RPE cells were treated with recombinant MeCP2 (Recombinant Protein (P01), Abnova, H00004204‐P01; 10 ng/mL, 72 hours), Recombinant TGF‐β (Peprotech, Rocky Hill; 10 ng/mL, 48 hours) or TNF‐α (R&D system, Minneapolis, MN; 20 ng/mL, 15‐39 minutesutes). The protein was extracted from the cells and subject to Western blot for the expressions of α‐SMA, PPAR‐γ and P‐MeCP2‐421 expression, respectively.

### 2.4 siRNA transfection

The RPE cells were cultured in 50% confluence condition. MeCP2 siRNA transfection was performed as previously publication (Li, et al, 2016). Briefly, the RPE cells were transfected with 10 nmol/L MeCP2 siRNA (2 hours) (stB‐0002766c) or scrambled siRNA (siN05815122147) (Guangzhou RiboBio Co., LTD) using HiPerFect Transfection Reagent (QIAGEN) as instructed by the manufacture. 48 hours after the transfection with or without TGF‐β (1‐5 ng/mL) treatment for additional 48 hours, the cells were harvested and protein was extracted from the cells and the expressions of Phosph‐Smad2/3, collagen I, FN and PPAR‐γ were analysed by Western blot.

### 2.5 Western Blot

The proteins from RPE cells were lysed using RIPA buffer and centrifuged at 12 000 ×g for 20 minutes, and protein concentration was determined by the Bio‐Rad protein assay kit (Bio‐Rad). Proteins were resolved on Tris‐HCl 4‐12% polyacrylamide gels at 110 V. The proteins were transferred to PVDF blotting membrane (Millipore, Bedford, MA). The membranes were blocked in 5% non‐fat milk and probed with antibody specific for Phosph‐Smad2/3 (Abcam), α‐SMA (Sigma‐Aldrich), Collagen1 (Biosis), FN (Abcam), PPAR‐γ (Biosis), P‐MeCP2‐421,80 and total MeCP2 overnight at 4°C. Membranes were washed and incubated with a horseradish peroxidase–conjugated secondary antibody (Vector Laboratories) for 30 minutes at room temperature. Images were visualized by addition of ECL chemiluminescence detection solution (Amersham Pharmacia Biotech). After stripping, the membranes were re‐probed with anti‐GAPDH antibody (Millipore) for protein loading control (Li, et al)^27^.

### 2.6 Chip assay

ChIP assay was performed using the Imprint Chromatin Immunoprecipitation Kit (Sigma‐Aldrich) according to the manufacturer's instructions. Chromatin from the RPE cells was first fixed with 1% formaldehyde for 10 minutes, and cells were fragmented using the Branson Sonifier (Branson). The RPE lysate was incubated with Protein A agarose (Sigma‐Aldrich) at 4°C for 45 minutes for pre‐clearing. The DNA‐protein complexes were then immunoprecipitated with rabbit anti‐MeCP2 antibody (Abcam) overnight at 4°C. DNA fragments were eluted by using DNA release solution and reversing solution provided by the kit. The resultant DNA including RPE samples and input was analysed by quantitative polymerase chain reaction (qPCR) and the TGF‐β2 primer sequences as follows: 5′‐CGGGAGACTTGATTGTCCTT‐3′ (sense) and 5′‐TTTGTTCCTGGATGACTCCC‐3′(anti‐sense). The PCRs were run using ZymoTaq Premix (Zymo Research, Irvine, CA) in the MyCycler Thermocycler (Bio‐Rad). The running conditions were 10 minutes at 95°C, followed by 35 cycles of 30 seconds at 95°C, 30 seconds at 56°C 1 and min at 72°C. PCR products were separated by electrophoresis on a 1.5% agarose gel.

## 3 RESULTS

### 3.1 P‐MeCP2‐421 and 80 expressions in PVR membranes

All the PVR membranes (10 patients, the average age was 38.9 years old) included in the study were positive for the expression of P‐MeCP2‐421 and 80 by immunohistochemistry analysis (Figure 1E, F); however, the intensity of the immunoreactivities of P‐MeCP2‐421 was much stronger than P‐MeCP2‐80 (Figure 1E). In contrast, the immunoreactivities of P‐MeCP2‐421 and 80 in normal retinal section were similar (Figure 1B and C).

**FIGURE 1:** P‐MeCP2‐421 and 80 expressions in representative human PVR membranes. (A, D) negative control, (B and C) immunohistochemical staining for P‐MeCP2 421, P‐MeCP2‐80 in normal retinal section (red chromogen) and blue for nuclear counter staining. Abundant P‐MeCP2‐421 expression was seen in PVR membrane (E), and the immunoreactivity of P‐MeCP2‐80 was similar in both normal retinal sections and human PVR membranes. Black arrows indicate positive MeCP2 staining. Original magnification, 400×

### 3.2 Co‐localization of P‐MeCP2‐421 with α‐SMA, cytokeratin, TGF‐β and PPAR‐γ in PVR membranes

Because we found that the expression of P‐MeCP2‐421 was dominated expressed in the PVR membranes, therefore, all double labelling was performed for the co‐localization of P‐MeCP2‐421 with the important molecules often to be seen in PVR membranes such as α‐SMA (Figure 2 A‐D), cytokeratin (Figure 2 E‐G), TGF‐β (Figure 3 A‐D) and PPAR‐γ (Figure 3 E‐H) in the PVR membranes. It was shown that α‐SMA, cytokeratin and TGF‐β were abundantly co‐localized with phospho‐P‐MeCP2‐421 in the PVR membranes, suggesting that many P‐MeCP2‐421‐positive cells derived from RPE and were trans‐differentiated. Interestingly, the immunoreactivity of PPAR‐γ was very low in the PVR membranes by the methods applied, and there was no obvious double labelling with P‐MeCP2‐421.

**FIGURE 2:** P‐MeCP2‐421 double labelling with α‐SMA (A‐D) and P‐MeCP2‐421 double labelling with cytokeratin (E‐G) in human PVR membrane. Localization of P‐MeCP2‐421 (red), α‐SMA (green) and cytokeratin (green) is shown in human PVR membranes. Yellow shows the double labelling of P‐MeCP2‐421 with α‐SMA or cytokeratin. Original magnification ×200

**FIGURE 3:** P‐MeCP2‐421 double labelling with TGF‐β2 (A‐D) and P‐MeCP2‐421 double labelling with PPAR‐γ (E‐H) in human PVR membrane. Localization of P‐MeCP2‐421 (red), TGF‐β2 (green) and PPAR‐γ (green) is shown in human PVR membranes. Yellow shows the double labelling of P‐MeCP2‐421 with TGF‐β2 or PPAR‐γ. Original magnification ×200

### 3.3 The effects of knocking down MeCP2 on the expressions of Phosph‐Smad2/3, collagen I, FN and the effects of recombinant MeCP2 on the expression of α‐SMA

Given P‐MeCP2‐421 is important for the pathogenesis of PVR, we then wanted to determine whether MeCP2 affects the important molecular that is recognized in the formation of EMT and fibrosis induced by TGF‐β. We found that knocking down MeCP2 by its specific siRNA inhibited the expression of Phosph‐Smad2/3 (Figure 4A), collagen I (Figure 5A) and FN (Figure 5B) induced by TGF‐β. The inactivation of Phosph‐Smad2/3 was especially striking after siRNA application. In addition, the expression of PPAR‐γ (anti‐fibrotic factor) was increased (Figure 5C), suggesting that MeCP2 was an important molecular for the induction of fibrosis induced by TGF‐β and plays an essential role in the pathogenesis of PVR. We did not detect significant cell death with the treatment of MeCP2‐specific siRNA or scrambled siRNA in the RPE cells under these conditions applied. Because knocking down MeCP2 could reduce the expression of α‐SMA,^21^ therefore, we determined whether α‐SMA would be affected by the supplement of exogenous MeCP2, as Western blot showed that α‐SMA expression increased by the stimulation of recombinant MeCP2 in the cultured RPE cells compared with control without MeCP2 addition (Figure 4. B), and the evidence further confirmed the role of MeCP2 in the mediation of EMT and fibrosis.

**FIGURE 4:** The effect of knocking down MeCP2 on the phospho‐Smad2/3 and the effect of recombinant MeCP2 on the expression of α‐SMA in the RPE cells. Knocking down MeCP2 inhibits expression of TGF‐β induced Smad2/3 activation as demonstrated by Western blot. The RPE cells were transfected with MeCP2 siRNA (+) or scrambled siRNA (−) 48 h with or without TGF‐β. GAPDH was used as protein loading control (A). Recombinant MeCP2 increased the expression of α‐SMA in the RPE cells as demonstrated by Western blot analysis. The RPE cells were treated with MeCP2 10 ng/mL or PBS 72 h and then subject to Western blot analysis. GAPDH was used as protein loading control (B)

**FIGURE 5:** The effect of knocking down MeCP2 using siRNA on the expressions of collagen I (A) and FN (B) and PPAR‐γ. The RPE cells were transfected with MeCP2 siRNA (+) or scrambled siRNA (−) 48 h with or without TGF‐β for additional 48 h, and then, the proteins were used for Western blot analysis. Knocking down MeCP2 inhibited expression of TGF‐β‐induced collagen I (A) and FN (B), but increases PPAR‐γ(C) as demonstrated by Western blot analysis. GAPDH was used as protein loading control

### 3.4 Binding of MeCP2 to TGF‐β

To confirm interaction of MeCP2 with TGF‐β gene in the RPE cells, specific antibody for MeCP2 antibody was used in a ChIP assay in the samples from the RPE cells. MeCP2 and TGF‐β complexes were immunoprecipitated. The eluted DNA from the immunoprecipitation was used for PCR magnification using TGF‐β promoter‐specific primer. As shown in Figure 6, a 465‐bp DNA fragment was amplified by PCR using the sample from MeCP2 antibody precipitated DNA, suggesting MeCP2 was bound to TGF‐β promoter in the RPE cells.

**FIGURE 6:** Chromatin immunoprecipitation (ChIP) was used to determine the interaction of MeCP2 and TGF‐β. MeCP2 and TGF‐β complex was immunoprecipitated using anti‐MeCP2 antibody. The eluted DNA from the immunoprecipitation was used for PCR magnification using a TGF‐β2‐specific primer. As the results showed that an expected PCR product for TGF‐β band was detected. 1. Molecular Markers. 2. no antibody CHIP (Negative control of CHIP assay); 3. MecP2 CHIP (with anti‐MeCP2 antibody); 4. Blank; 5. Total input (positive control); 6. Negative control (no template)

### 3.5 The effects of TGF‐β on the expression of PPAR‐γ expression

There were abundant immunoreactivity of PPAR‐γ in the RPE cells without TGF‐β addition; however, the treatment of the RPE cells with TGF‐β (10 ng/mL) inhibited the expression of PPAR‐γ as shown in Figure 7A by Western blot, and PPAR‐γ protein was reduced even at the concentration of 5ng/ml of TGF‐β, up to 10 ng/mL of TGF‐β treatment on PPAR‐γ was almost undetectable (Figure 7. A). On the other hand, treatment of the RPE cells with MeCP2 inhibitor 5‐AZA increased PPAR‐γ expression (Figure 7B). Figure 7C showed the relevance of reduction of PPAR‐γ to MeCP2 by immunofluorescent staining, and it was demonstrated that silence of MeCP2 by siRNA increased the expression of PPAR‐γ, suggesting that PPAR‐γ expression was under the regulation of MeCP2.

**FIGURE 7:** The effect of the expression of PPAR‐γ by TGF‐β (A), 5‐AZA (B) and siRNA MeCP2 (C) in the RPE cells. TGF‐β inhibits the expression of PPAR‐γ, and the strongest inhibition can be seen at the concentration of 10ng/ml of TGF‐β(A); however, PPAR‐γ expression is up‐regulated by the treatment of 5‐AZA up to 2µM(B); knocking down MeCP2 using siRNA results in an increased expression of PPAR‐γ as shown by immunocytochemistry (C)

## 4 DISCUSSION

MeCP2 is critically important for normal cell function maintaining, and abnormal expression of MeCP2 is related to many pathologic conditions including EMT and fibrosis.^19^, ^21^, ^22^, ^28^, ^30^ The expression of non‐phosphorylated MeCP2 in numerous fibrotic tissue such as liver,^19^, ^22^ lung,^24^ heart ^23^ and PVR membranes ^21^ has been reported. Here, we determined that the expression of P‐MeCP2‐421 and MeCP2‐80 expressions in human PVR membranes as demonstrated by immunohistochemistry, although the staining of both MeCP2‐421 and MeCP2‐80 was positive in the PVR membranes, the immunoreactivity of P‐MeCP2‐421 was considerably stronger than 80, and there was no obvious difference of the expression of P‐MeCP2‐421 and MeCP2‐80 between normal retinal section and PVR membranes; therefore, P‐MeCP2‐421 was chosen for the rest of double labelling.

Phosphorylation is an essential of cellular signalling event; P‐MeCP2‐421 is one of MeCP2 phosphorylation. Our results showed that P‐MeCP2‐421 co‐localized with cytokeratin (imply RPE cells), α‐SMA (trans‐differentiated cell) and TGF‐β in PVR membranes. It is known that phosphorylation of MeCP2‐421 leads to dissociation of sin3, HDAC and MeCP2 from a transcription repress to be a gene activator,^31^ and it is possible that the increased expression of those fibrotic molecules such as α‐SMA and TGF‐β in PVR might be mediated by MeCP2 phosphorylation at Serin421.^31^ The differentiation of the expression of P‐MeCP2‐421 and P‐MeCP2‐80 in term of gene silence or activation has been reported previously.^34^, ^35^ Phosphorylated MeCP2‐421 and MeCP2‐80 are the two major event in keeping homeostasis of cell function under normal condition that is called Yin and Yang.^34^, ^35^ It is shown that inhibition of phosphorylated MeCP2‐80 increased neuronal activity, and MeCP2‐80 phosphorylation reduced hepatic stellate cells proliferation and liver fibrosis ^36^; in contrast to MeCP2‐80 phosphorylation, the neuronal activity and gene activation are associated with phosphorylation of MeCP2‐421.^34^, ^37^ In our study, the increased P‐MeCP2 421 instead of P‐MeCP2‐80 was seen in the human PVR membranes; more likely, the balance between P‐MeCP2‐80 and P‐MeCP421 was lost in the process of development of PVR.^35^, ^37^ Therefore, the highly expressed P‐MeCP2‐421 may play an important role in the pathogeneses of PVR.

It is well recognized that TGF‐β is a major inducer of fibrosis in retina and systemic diseases. We found that P‐MeCP2‐421 was preferentially expressed in PVR membranes and was double labelled with TGF‐β to demonstrate the effects of the MeCP2 on TGF‐β‐induced downstream gene products would be interesting; therefore, we looked into if knockdown MeCP2 could alter activation of TGF‐β signalling especially its downstream Smad2/3 activation (the major signalling of TGF‐β). As the result shown in Figure 4 A, TGF‐β treatment alone caused the expected activation of Smad2/3. In contrast, when the cells were transfected with MeCP2 siRNA, the Smad2/3 activation induced by TGF‐β was inhibited. Because the suppression of Smad2/3 activation by MeCP2 siRNA, a strong inhibition of the expression of collagen I and FN, which are the downstream fibrotic genes of TGF‐β and the important components in fibrotic PVR membranes, was also demonstrated. The results suggested that TGF‐β signalling might be subject to MeCP2 regulation, although TGF‐β signalling activation is regulated by multiple factors and is complex.

The critical phenotype of epithelial cell trans‐differentiation including RPE is the increased expression of α‐SMA. α‐SMA is a marker of EMT and is rich in the fibrotic tissue. TGF‐β is the major inducer of α‐SMA expression. We found that both α‐SMA and P‐MeCP2‐421 were highly expressed and double labelled in PVR membranes, indicating the importance of MeCP2 in the mediation of fibrosis. We then investigated into the direct effects of MeCP2 on the expression of α‐SMA in the RPE cells; as the result shown in Figure 4B, stimulation of the RPE cell with recombinant MeCP2 leaded to the up‐regulation of α‐SMA, and the founding was similar to the result that transfection with MeCP2 plasmid enhanced α‐SMA expression in fibroblast,^24^ but we expanded previous study by using recombinant MeCP2 in the RPE cells. The notion that MeCP2 could regulate α‐SMA expression is further validated, it is found that without MeCP2 the expression of α‐SMA is greatly diminished,^38^ and the reason of the up regulation of α‐SMA by MeCP2 is because MeCP2 can binds to α‐SMA gene and enhance α‐SMA expression.^24^ Taken together, MeCP2 might be an enhancer of α‐SMA expression and participates in the formation of fibrosis and PVR.

As both P‐MeCP2‐421 and TGF‐β are rich in PVR membranes, therefore we asked if there is an interaction between MeCP2 and TGF‐β in the RPE cell, a ChIP assay was performed using anti‐MeCP2 antibody and then DNA from the protein‐DNA complex was amplified by human TGF‐β2 primer. As seen in Figure 6, a DNA fragment (∼456 bp) for TGF‐β was demonstrated. No band was detected when control IgG was used, indicating specific precipitation by the anti‐MeCP2 antibody. Moreover, no band was detected when template was not used. The observation of MeCP2 binding to the TGF‐β gene promoter implied the function interaction between two molecular and knocking down MeCP2 compromised TGF‐β signalling as mentioned previously, suggesting that MeCP2 plays a critical role in TGF‐β‐induced EMT/fibrosis.

One of important phenomenon in the formation of fibrotic tissue is the reduction of PPAR‐γ,^18^, ^19^, ^22^, ^39^, ^40^ and decreased expression of PPAR‐γ is seen in numerous systemic fibrotic diseases, implying that there is the loss of PPAR‐γ in the process of fibrotic tissue formation.^18^, ^19^, ^22^, ^39^, ^40^ The rational for us to study PPAR‐γ was because in the current study, we found that the expression of PPAR‐γ in PVR membranes was extremely low. It was almost under detectable in methods applied and diminished PPAR‐γ protein expression, and elevated levels of MeCP2 transcript were revealed in the PVR membranes; further, the expression of PPAR‐γ was inhibited in the RPE cells by the treatment of TGF‐β, importantly, knocking down MeCP2 by siRNA and the addition of a MeCP2 inhibitor 5‐AZA in the cultured RPE cells, and the expression of PPAR‐γ was up‐regulated. Our result is supported by previous publication by Mann et al in which the silence of PPAR‐γ in the fibrotic tissue of liver is associated with highly expressed MeCP2 ^19^, ^22^; more likely, one mechanism by which MeCP2 mediated the fibrosis process in PVR may be through the inhibition of PPAR‐γ.^22^

In summary, our study demonstrates a novel role of P‐MeCP2‐421 in retinal fibrosis specifically in the pathogenesis of PVR and identifies critical intracellular targets (such as α‐SMA, Sm ad2/3, collagen I, FN, PPAR‐r) in the formation of fibrosis that is regulated by MeCP2, suggesting MeCP2 could be potentially targeted for therapy in the treatment of PVR and other fibrotic diseases.

## CONFLICT OF INTERESTS

All authors declare that no competing interests exist.

## AUTHOR CONTRIBUTIONS

**Xiaohua Li:** Conceptualization (lead); Data curation (lead); Funding acquisition (lead); Investigation (lead); Methodology (lead); Supervision (lead); Writing‐original draft (lead). **Xue Li:** Data curation (equal); Investigation (equal). **Shikun He:** Conceptualization (equal); Data curation (equal); Supervision (equal); Writing‐original draft (equal). **Mingwei Zhao:** Conceptualization (equal); Data curation (equal); Supervision (equal); Writing‐original draft (equal).

## Data Availability

All data were included in the manuscript.
